# Clinical application of 675 nm laser therapy for dorsal hand skin hyperpigmentation

**DOI:** 10.1111/srt.13484

**Published:** 2023-10-04

**Authors:** Ido Alter, Irene Fusco, Francesca Madeddu, Tiziano Zingoni

**Affiliations:** ^1^ Private Clinic Tel Aviv Israel; ^2^ El.En. Group Calenzano Italy

**Keywords:** 675 nm laser therapy, clinical evidence, photodamaged hands, skin hyperpigmentation

## Abstract

**Background:**

Noninvasive skin rejuvenation treatment is growing in recognition to aesthetic medicine.

**Aim:**

The objective of the study was to assess the efficacy and the safety of the 675‐nm laser source treatment of photodamaged hands.

**Materials and methods:**

The study included 21 patients (6 males and 15 females) with a mean age of 63 (± 9) years. Patients were treated with —two to three sessions of the 675‐nm laser with a 1‐month interval between sessions. Photos of each patient were collected at baseline, and 3 months after the last laser session. The 5‐point Global Aesthetic Improvement Scale (GAIS) was recorded with their final assessment session (3 months).

**Results:**

The total GAIS scores showed satisfactory results: 15 patients (71%) experienced 4 score (excellent improvement) changes and 6 patients (29%) experienced 3 score (good improvement) changes. Clinical images showed good efficacy and visible aesthetic results for the management of photodamaged skin. No serious adverse effects were recorded.

**Conclusion:**

This study demonstrates the safety and efficacy of for the aesthetic improvement of skin pigmentation and texture for photodamaged hands.

## 1 INTRODUCTION

Hyperpigmentation, whether localized or generalized, is frequent in dermatology.^1^, ^2^, ^3^ There are numerous causes, and determining the aetiology is often difficult.

Skin hyperpigmentation, a common dermatological condition, causes the skin's colour to typically darken. According to Pérez‐Bernal et al.,^4^ a number of internal and external factors, such as hormonal changes, inflammation, injury, acne, eczema, certain medications or UV exposure, can cause these changes in skin coloration. The biological processes that result in the production of the skin pigment melanin by melanocytes in various layers of skin determine the pigmentation and coloration of the skin. Thus, disorders of skin hyperpigmentation are caused by changes in melanocyte production or melanin distribution.^5^

The need and demand for newer, safer, and more efficient treatments for different hyperpigmentation conditions has made it possible for researchers to continuously investigate treatment options.

Non‐invasive skin rejuvenation treatment is growing in recognition to aesthetic medicine, with novel techniques now targeting aging hands, a cosmetic indication that extends beyond the more traditional aging face and decolletage indications. With non‐invasive procedures for facial rejuvenation becoming increasingly effective in recent years, a patient's true age is becoming visible on the hands, creating an interest for and desire for efficient therapies in this area.

It is becoming more common to use ablative and non‐ablative energy‐based devices for the cosmetic improvement of aging hands, which are typically characterized by the development of dyschromias, fine telangiectasias, solar lentigines/keratoses and a progressive loss of skin texture/atrophy resulting in varying degrees of wrinkling, fine lines, and skin laxity occurring as a result of both intrinsic and extrinsic aging processes.^6^, ^7^

For the medical management and cosmetic improvement of photo‐aged skin, a variety of minimally and non‐invasive therapies are currently available. These methods range from the injection of neurotoxins and a wide variety of filler products with different compositions, topical agents, chemical peels, oral therapies, to the use of energy‐based modalities like focused ultrasound, RF, laser, and light‐based technologies. However, the use of the majority of these current treatment modalities, especially peels or ablative devices, is restricted due to unwanted side effects such as post inflammatory hyperpigmentation (PIH), prolonged downtime, low treatment tolerability and risk of scarring.^8^, ^9^

The application of topical substances, such as hydroquinone‐based preparations, have been used for a long time in order to improve the cosmesis of pigmented lesions. However, they are insufficiently effective in the treatment of solar lentigines and, furthermore, they fail to treat other aspects of photo‐aging, such as wrinkles, fine lines and skin hyperpigmentation. Chemical peels come next as second‐line treatment, which have shown good efficacy but poses a greater risk of side effects and is more expensive. Oral therapies have usually demonstrated mixed results and more relapse rate.^10^

Furthermore, hand rejuvenation has been related to a higher risk of side effects compared to facial rejuvenation. Since hand skin is thin and has few pilosebaceous units, wound healing is slow and scarring is more prevalent.

Thus, only low energies of energy‐based devices can be used in this area.

RF‐based devices and intense pulsed light (IPL) technology have become very popular in skin rejuvenation therapy due to the excellent treatment outcomes achievable coupled with minimal downtime, a favourable safety profile and a high tolerability associated with the noninvasive treatment approach.^7^, ^11^ Furthermore, due to the nature of the delivery of heat energy to the skin, the use of RF in skin rejuvenation procedures has been shown to be safe and effective in individuals with darker phototypes.^12^ The application of optical energy in the form of intense pulsed light (IPL), a wide‐spectrum light source, has long been considered an efficient and secure approach for the management of solar lentigines, skin rejuvenation and photodamaged skin.^11^, ^13^

Especially, the wavelength of 675 nm has proven to be an effective and safe laser source system for skin ageing^14^, ^15^, ^16^, ^17^, ^18^ and hyperpigmented disorder management in both for light and dark skin types as reported in literature.^19^, ^20^

However, in view of the success obtained with 675 nm laser treatment for skin rejuvenation and hyperpigmented disorder, its effect has never been clinically tested for dorsal hand skin hyperpigmentation. Therefore, the innovative aspect of the current research was to show a different application and a different mechanism of action of the 675 nm laser in a new body area using different and specified protocol.

For this reason and on the basis of previously validated scientific findings, the current study evaluates the efficacy and the safety of the 675‐nm laser source cosmetic treatment for the improvement of hyperpigmentation and photo‐damaged skin on the back of the hands, which represented a high‐risk area for the onset of photodamaged sings.

## 2 MATERIALS AND METHODS

### 2.1 Device description

All subjects were treated with the RedTouch laser system (DEKA M.E.L.A, Italy). The study device emits a wavelength of 675 nm and it is equipped with a 13 × 13 mm scanning system with a contact sensor, integrated in the handpiece, able to generate fractional micro‐zones of 0.7 mm width (DOT) of either sub‐ablative and selective thermal damage on the skin preserving the epidermal layer thanks to an integrated skin cooling system, which protect the health of the skin while minimizing downtime.

### 2.2 Patient population and study design

The study included 21 patients (6 males and 15 females) with a mean age of 63 (± 9) years old (age ranged between 42 and 74 years). Fifteen patients presented Fitzpatrick skin type II and 6 patients presented Fitzpatrick skin type III.

Exclusion criteria for the study were the following: patients hypersensitive to light in the near‐infrared wavelength region, the use of photosensitizing agents, the use of anticoagulant and/or immunosuppressant, patients with seizure disorders triggered by light, pregnant patients, patients with personal or family history of skin cancer, patients exposed to the sun during the 3 weeks before treatment, the presence of tattoos or skin disorders on the treated areas.

Patients were treated with —two to three sessions of the 675‐nm laser with a 1‐month interval between sessions. The following laser parameters were selected: power 7–10 W, dwell time 75 ms, spacing 0 μm and Energy/DOT 525 – 750 mJ/DOT.

Before starting the treatment, areas to be treated were cleaned with a mild soap and rinsed with water. The energy treatment assessment was carried out for each patient on a dedicated area “test” based on the subject's skin type and degree of tolerability. The answer to the test was noticeable within 48/72 h. The endpoint was considered a darkening of the treated lesion. The treatment was performed by positioning the handpiece perpendicular to the lesion to be treated. For each lesion, the shape and size of the scan area was modified to hit only the desired target. After treatment, the skin was cooled with gauzes soaked in cold water and a moisturising emulsion to the skin was applied.

### 2.3 Outcomes assessment

For documentation, photos of each patient were collected. Standardized Clinical photographs were acquired using a digital camera (Reflex Nikon D800, Nikon Corporation, Minato, Tokyo, Japan) at baseline, and 3 months after the last laser session. The 5‐point Global Aesthetic Improvement Scale (GAIS) (0 point—no change; 1 point ‐ 25% mild improvement; 2 points ‐ 50% moderate improvement; 3 points −75% good improvement; 4 points‐ 100% excellent improvement) (Table 1) was recorded at their final assessment session (3 months). The GAIS is a validated scale and a generalized aesthetic qualitative assessment by the observer for assessing changes in skin texture and pigmentation. This scale also allows an assessment to be made of patient satisfaction with treatment, an important (though highly subjective) outcome.^21^ Before starting the laser treatment, every subject provided their written informed consent.

**TABLE 1:** The 5‐point Global Aesthetic Improvement Scale scores.

5‐Point GAIS	Improvements
0 point	No change
1 point	25%—mild improvement
2 points	50%—moderate improvement
3 points	75%—good improvement
4 points	100%—excellent improvement

### 2.4 Side effects

Adverse events such as oedema, burns, formation of keloids, excessive pain, crusting, scars, prolonged erythema, blisters or dyschromia were evaluated at the post‐treatment visit.

## 3 RESULTS

All patients completed the study. On the basis of investigator‐evaluated GAIS scale, the total GAIS scores showed satisfactory results: As reported in Figure 1, 15 patients (71%) experienced 4 score (excellent improvement) changes and 6 patients (29%) experienced 3 score (good improvement) changes. None of the patients experienced no change, mild improvement or moderate improvement.

**FIGURE 1:** Physician assessment of improvement for laser treatment at 3‐month follow‐up visit.

Clinician assessment from the clinical photography showed good improvement in hand pigmentation, skin texture and laxity.

One of the clinical cases with good aesthetic results is represented in Figure 2.

**FIGURE 2:** Female patient with pigmentation and photo‐aged hands before (A) and 3 months after laser treatment (B).

No serious adverse side effects were recorded. The only side effect is a mild sensitivity that resolve in 2–3 h after the treatment.

## 4 DISCUSSION

Hyperpigmentation is not considered a harmful or lethal disorder; however, it can affect the quality of life of patients by affecting their emotional and psychological health.

Light‐based therapies have been proven to influence and perhaps reverse skin ageing at clinical, molecular and histologic levels. Particularly, 675 nm laser technology decreases photodamage by promoting collagen type I and III synthesis and enhancing the expression of heat shock protein, as demonstrated by a recent study^17^ which showed that various 675 nm radiation doses have potential therapeutic benefits on the process of skin rejuvenation in human dermal fibroblast cells.

In another recent published study,^22^ the 675 nm laser technology was also found to be safe and effective in treating facial melasma. However, despite it represents the same laser technology, in our study a different protocol on a different anatomical location was applied than the one used for the treatment of melasma. Indeed, in this paper the clinical application was different. In the previously published article,^22^ the 675 nm laser was shown to be effective in treating facial melasma, but the dermatological condition being treated in the current study is a dorsal hand skin hyperpigmentation for which a 675 nm laser treatment has never been clinically tested.

Therefore, the innovative aspect of the current research was to show a different application and a different mechanism of action of the 675 nm laser in a new body area using different and specified protocol.

Based on the results of the current study and those already present in the literature, we demonstrated that treatment with a wavelength of 675 nm for skin rejuvenation not only leads to a better clinical improvement of the pigmented lesion with a very low risk of side effects, but also allows for a remarkable tissue tightening and textural improvement of the skin surface. Furthermore, we chose a high‐risk area such as the hands for this study to be able to effectively demonstrate the efficacy and safety of this new 675 nm wavelength technology. At 3 months follow‐up with investigator assessments, pigmentation and skin laxity were marked improved in the hands treated with 675 nm wavelength; indeed, the total GAIS scores showed satisfactory results with any discomfort for the patients, which are confirmed also by the photographic evaluation.

The treatment strategy produced a more thorough skin rejuvenation of the back of the hands, including the lightening and clearing of pigmented lesions as well as a visibly noticeable improvement in the smoothness and laxity of the skin with minimal procedural downtime.

This study represents the first clinical investigation that examines the impact of the 675 nm wavelength on dorsal hand skin hyperpigmentation, which is one of the most at‐risk areas due to its excessive sun exposure.

Our study's limitation is the small number of patients. Our long‐term goal is to increase the number of patients treated, as well as to extend follow up period.

## 5 CONCLUSION

This study demonstrates the safety and efficacy of 675 nm laser system for the aesthetic improvement of skin pigmentation and texture for photodamaged hands.

## CONFLICT OF INTEREST STATEMENT

Irene Fusco, Francesca Madeddu and Tiziano Zingoni are employed at El.En. Group. The other authors declare that the research was conducted in the absence of any commercial or financial relationships that could be construed as a potential conflict of interest.

## Data Availability

On reasonable request, the corresponding author will provide the information supporting the study's results.
